# Resveratrol as a Promising Polyphenol in Age-Associated Cardiac Alterations

**DOI:** 10.1155/2022/7911222

**Published:** 2022-06-18

**Authors:** Denise Börzsei, Judith Sebestyén, Renáta Szabó, Zelma Nadin Lesi, Andrea Pálszabó, Patrícia Pálszabó, András Szász, Dániel Priksz, Béla Juhász, Médea Veszelka, Zsolt Turcsán, Zoltán Deim, Csaba Varga, Anikó Pósa

**Affiliations:** ^1^Department of Physiology, Anatomy and Neuroscience, Faculty of Science and Informatics, University of Szeged, 6726 Szeged, Hungary; ^2^South-Pest Hospital Centre, National Institute for Infectology and Haematology, Department of Burns and Plastic Surgery, Budapest 1097, Hungary; ^3^Institution of Physical Education and Sport Sciences, Faculty of Education, University of Szeged, 6725 Szeged, Hungary; ^4^Department of Pharmacology and Pharmacotherapy, Faculty of Medicine, University of Debrecen, 4032 Debrecen, Hungary; ^5^Gulyás János és Társa Ltd., 6645 Felgyő, Hungary

## Abstract

According to a widely accepted theory, oxidative stress is considered to be the number one trigger of aging-associated degenerative processes including cardiovascular diseases. In the context of aging-research, resveratrol receives special attention with its surprising number of health benefits. The aim of our study was to examine the anti-inflammatory and antioxidant effects of this dietary polyphenol in aging rat heart. 20-month-old female and male Wistar rats were divided into control (untreated) and resveratrol-treated groups. Resveratrol was administered at a dose of 0.05 mg/ml for 12 weeks dissolved in drinking water, while the control rats received *ad libitum* water. Cardiac level of reactive oxygen species (ROS), nuclear factor kappa B (NF*κ*B), tumor necrosis factor alpha (TNF-*α*), and glutathione (GSH) parameters, as well as the activity of myeloperoxidase (MPO) and heme oxygenase (HO) enzymes were detected. Together with the biochemical measurements, hearts were isolated and used for an exposure of ischemic-reperfusion injury via Langendorff perfusion system. 12 week of resveratrol treatment suppressed the age-related inflammatory pathways including the expression of TNF-*α*, NF*κ*B, and the activity of MPO while intensified the endogenous antioxidant defenses through the induction of GSH and HO system. Presumably, as a result of these processes, the necrotic area of the heart in response to an acute injury was also significantly reduced in the resveratrol-treated groups. Our findings confirmed that resveratrol has cardioprotective effects at several points by counteracting the aging-associated cellular malfunctions in the heart.

## 1. Introduction

Aging is a multifactorial biological process driven by a variety of cellular changes which ultimately affect protein homeostasis, chromosome structure, and genetic information. The hallmarks of aging are postulated to originate from oxidative damages and the resulting disrupted redox imbalance [1]. Oxidative stress can cause premature apoptosis or senescence by impairing the cellular milieu, and this altered cellular fate serves as a major determinant of lifespan [2]. Furthermore, it is important to note that changes in cellular redox status and cell death signaling pathways are also causally related to the development of chronic inflammation [3]. Age-related oxidative stress and inflammation inevitably pose a threat to cardiovascular health; however, with the latest medical advancements, antioxidant active agents, and lifestyle changes, it is now possible to slow down aging processes and avert the progression of age-related cardiovascular conditions [4–6].

Resveratrol (RESV) is a stilbenoid polyphenol originally extracted from the roots of *Veratrum grandiflorum* but has been detected in many other plants since then, such as grapes, berries, and peanuts. It exists in two isoforms, namely, *cis-, trans*-resveratrol, the latter of which is considered to be a more biologically active and stable form [7]. In 1992, Renaud and De Lorgeril were the first who set a parallel between wine-related polyphenols and reduced risk of adverse cardiovascular outcomes and named this phenomenon the “French paradox” [8]. RESV has gained an outstanding scientific interest ever since due to its wide-ranging biological effects. It has a remarkable ability to counteract a number of noncommunicable diseases and has been shown to be particularly effective in the treatment of cardiovascular diseases (CVD) thanks to its anti-inflammatory and antioxidant properties. [9–11]. Numerous experimental studies verified that RESV plays an important role in the prevention of CVDs by affecting cardiac Ca^2+^ homeostasis, hypertrophic signaling pathways, and myocyte apoptosis [12–14]. Additionally, it has also been demonstrated that RESV has an exceptional capability to extend the lifespan of multiple model organisms, bolstering hope that these findings can be translated into further medical studies in the future [15].

Based on the literature, we assumed that a long-term RESV intake may be an effective agent against age-derived myocardial damages in rat model. Therefore, the aim of our study was to explore the cardiac anti-inflammatory and antioxidant effects of RESV and whether these RESV-mediated protective effects are manifested in acute cardiac injury.

## 2. Materials and Method

### 2.1. Experimental Protocol

In this study, 20 month-old male and female Wistar rats (*n* = 7 − 9 rats per group) were used (Toxi-Coop, Hungary). Animals were kept under standard circumstances according to the regulations of the Directive 2010/63/EU. At the beginning of the study, within the sexes, rats were divided into the following two subgroups: control (CTRL) and RESV-consuming animals. Control rats received *ad libitum* water throughout the study, while RESV animals got 0.05 mg/ml*trans*-resveratrol (AK Scientific, USA) dissolved in their drinking water for 12 weeks [16]. This dose was chosen to provide the adequate mg/kg bodyweight dose (7.5 mg/kg) based on the animals' consumption [17]. Dissolved RESV was placed into the cages in a tinted glass in order to prevent photochemical isomerization. At the end of the study, rats were sacrificed, and their hearts were either perfused via Langendorff system in order to expose the size of infarction as a result of a left anterior descending coronary artery (LAD) occlusion or were clamped and stored at -80°C for further biochemical measurements. All procedures were approved by the National Scientific Ethical Committee on Animal Experimentation (XX./2317/2021.) and correspond to the ARRIVE guidelines.

### 2.2. Ischemia-Reperfusion Injury Modelling with Langendorff Perfusion System

After anesthesia, animals were subjected to cervical dislocation, and their hearts were removed by maximal aortic excision. Using an ice-cold Krebs-Henseleit buffer (1.24 mM KH_2_PO_4_, 20.1 mM NaHCO_2_, 1.25 mM CaCl_2_, 4.7 mM KCl, 119 mM NaCl, 1.24 mM MgSO_4_, 11.2 mM glucose, and 1.24 mM MgSO_4_), hearts were suspended through the aorta and placed on a Langendorff perfusion column. Retrograde perfusion of the hearts was performed under the following conditions: pressure 75 mm Hg, 5% CO_2_, 95% O_2_, and 37°C. Ischemic injury was modeled by LAD ligation for 30 min followed by reperfusion for 120 min. Hearts were then perfused with Evans blue solution (1%) and placed in a -20°C freezer until further analysis.

### 2.3. Determination of Infarct Size

To determine the area of infarct, frozen hearts were sliced into 2 mm-thick pieces perpendicular to the apico-basal axis and incubated at 37°C for 10 min in 1% 2,3,5-triphenyl tetrazolium chloride (TTC) solution. Slices were then immersed in 10% formalin solution and washed with phosphate buffer (pH 7.4). The heart slices were photographed between two glass slides, and the infarction area was evaluated using Image J program, its size was expressed as the percentage of the area at risk.

### 2.4. Determination of NF*κ*B, ROS, and TNF-*α* Concentration

Powdered heart tissues were homogenized with a given amount of phosphate-buffered saline (PBS; pH 7.4) with a handheld homogenizer. Samples were placed in the centrifuge for 20 minutes (at 2000 rpm, 4°C); then, supernatants were collected and kept on ice. Standards were diluted according to the manual of the Enzyme-linked Immunosorbent Assay (ELISA; GenAsia Biotech) kits. Sample solution wells included 40 *μ*l sample, 10 *μ*l antibody, and 50 *μ*l streptavidin-HRP. After covering the plate with a seal plate membrane, reagents together with samples were incubated at 37°C for 60 minutes. Color development was initiated by chromogen solutions A and B and stop solution. At the end of the assay, absorbance (OD) of each well was measured under 450 nm wavelength. The color shade of the samples is positively correlated with the concentration of the aforementioned enzymes. NF*κ*B and TNF-*α* values were defined as pg/mg protein, while ROS concentration was expressed as *μ*U/mg protein.

### 2.5. Determination of MPO Activity

Heart tissues were homogenized twice for 10 seconds in a buffer containing PBS and 0.5% hexadecyltrimethylammonium bromide (HETAB). Samples were frozen and thawed four times, for better cell disruption; then, homogenates were centrifuged for 15 minutes, at 10 000 and 4°C. For the activity measurement, 12 *μ*l of standard or sample was added to a 96-well plate, followed by 280 *μ*l of o-dianisidine dihydrochloride. The reaction was started with 20 *μ*l of hydrogen peroxide, and after shaking the reaction mixture for 30 seconds, the activity of MPO was detected spectrophotometrically at 490 nm. The values were expressed as *μ*U/mg protein.

### 2.6. Determination of Total GSH+GSSG Content

Rat hearts were first homogenized on ice in a buffer [0.25 M sucrose, 20 mM Tris, and 1 mM dithiothreitol (DTT)], and the resulting homogenate (15 000 g, 30 min, 4°C) was centrifuged. From the supernatant obtained after centrifugation, 1 ml was further homogenized with 200 *μ*l of homogenization buffer (0,25 M sucrose, 20 mM Tris, 1 mM DTT, and 0,1 M CaCl_2_). After incubation on ice for 30 min, another centrifugation was performed (21 000*g*, 30 min, and 4°C). The resulting pure cytosolic fraction was used for enzyme assay. In a 96-well microplate, 40 *μ*l of sample or standard, 20 *μ*l of 5,5′-dithio-bis-2-nitrobenzoic acid, and 140 *μ*l of nicotinamide dinucleotide phosphate (NADPH) were added, and the resulting mixture was incubated for 5 min at 25°C. The reaction was started by adding 10 *μ*l of glutathione reductase. After shaking for 10 min, the formation of 2-nitro-5-thiobenzoic acid was measured at 405 nm, and the resulting GSH levels were expressed as nmol/mg protein.

### 2.7. Measurement of HO Activity

Cardiac tissues were homogenized in ice-cold buffer (10.0 mM N-2-hydroxyethylpiperazine-N'-2-ethanesulfonate, 0.10 mM ethylenediamine-tetraacetic acid disodium salt dihydrate, 1.0 mM DTT, 30.0 mM sucrose, 10 *μ*g/ml trypsin inhibitor, 2.0 *μ*g/ml aprotinin, 10.0 *μ*g/ml leupeptin, and pH 7.4), centrifuged at 15 000×*g*, for 20 min, at 4°C, and the remained supernatant was used for HO activity measurements. The reaction mixture consisted of 75 *μ*l of sample, 2.0 mM glucose-6-phosphate, 0.14 U/ml glucose-6-phosphate dehydrogenase, 15.0 *μ*M hemin, and 120.0 *μ*g/ml biliverdin reductase. For the determination of HO activity, two parallel measurements were performed, a so-called blind and NADPH line. For the NADPH measurement, 100 *μ*l of reduced *β*-nicotinamide adenine dinucleotide phosphate (*β*-NADPH) was added to the mixture to initiate the reaction and incubated at 37°C for 60 min, after which ice cooling was used to stop the reaction. For the blank measurements, a reaction mixture was prepared in which *β*-NADPH was replaced with buffer. The NADPH and blank solutions were measured spectrophotometrically at 465 nm; the values obtained from the blank series were then subtracted from the NADPH values. HO activity was plotted as the amount of bilirubin formed in nmol/hour/mg protein.

### 2.8. Measurement of Protein Concentration (Bradford Method)

In order to perform the protein measurements, the samples which were homogenized and centrifuged according to the previous measurements had to be diluted appropriately in parallel with the preparation of a new standard line. After the dilution, 200 *μ*l of Bradford reagent was added to both the standard bovine serum albumin (BSA) line and our samples. The protein concentration of the samples was measured at 595 nm by a spectrophotometer, results were expressed at *μ*g protein/ml.

### 2.9. Data Representation and Statistical Analysis

Experiments were designed to generate groups of equal size using randomization. Group sizes represent the number of independent samples/animals, not technical replicates. Raw data was analyzed by a blinded reader. Data presented as the mean value of the group ± standard deviation (mean ± SD). Normal distribution was estimated by Shapiro-Wilk normality test; after, statistical analysis was performed using one-way analysis of variance (ANOVA) followed by Tukey posttest (only if *F* in ANOVA achieved *p* < 0.05, and normality test was passed) or Kruskal-Wallis test followed by Dunn's posttest (when normality test was not passed). Statistical analysis was performed using the GraphPad Prism 8.4.2. (GraphPad Software Inc., La Jolla, CA, USA; RRID:SCR_002798). Probability values (*p*) less than 0.05 were considered significantly different; and the level of significance is marked with asterisks between the corresponding groups (^∗^: *p* < 0.05; ^∗∗^: *p* < 0.01; ^∗∗∗^: *p* < 0.001; ^∗∗∗∗^: *p* < 0.0001).

## 3. Results

### 3.1. Measurement of Myocardial Infarct Size

As shown in Figure 1, aging CTRL animals have shown a higher rate of infarct size compared to the RESV-treated groups. As a result of the 12-week-long RESV consumption, a significant attenuation was detected in the necrotic extension of the heart in both sexes.

### 3.2. Cardiac TNF-*α* and NF*κ*B Concentration

Members of the inflammatory cascade, namely, TNF-*α* and NF*κ*B concentrations, were markedly elevated in aging CTRL groups compared to the RESV groups. 12 weeks of RESV administration was able to significantly mitigate these elevated proinflammatory values in both females and males. Data are presented in Figures 2(a) and 2(b).

### 3.3. Cardiac MPO Activity

Figure 3 presents that similar to the inflammatory TNF-*α* and NF*κ*B expression, CTRL aging female and male rats exhibited the highest MPO activities; whereas 12 weeks of RESV administration resulted in a decreased MPO activity in both sexes; furthermore, in females, this change was found to be significant.

### 3.4. Cardiac ROS Concentration

As shown in Figure 4, aging status resulted in a marked increase in the ROS expression of male and female rats. Nonetheless, for both sexes, RESV-treated rats possessed significantly lower ROS values in comparison with the CTRL animals.

### 3.5. Determination of Cardiac Total GSH+GSSG Content

As a result of the 12-week RESV treatment, a significant improvement was detected in the cardiac antioxidant status in both male and female aged rats. As for female rats, GSH+GSSG content alteration in response to the RESV administration was found to be significant. Data are presented in Figure 5.

### 3.6. Measurement of Cardiac HO Activity

As shown in Figure 6, RESV-consuming animals exhibited the highest HO activity values, whereas a significant decrease was found in CTRL aging animals; thus, the reduced antioxidant values precipitated by aging were compensated by 12 weeks of RESV treatment.

## 4. Discussion

The quest to discover the secret of longevity has been on-going for quite some time. It is apparent that life expectancy and cardiovascular aging are closely interrelated, both from a cause-and-effect perspective and from a prevalence point of view [2]. Based on the most widely accepted theories today, the primary cause of aging is the accretion of ROS and the resulting accumulative oxidative damage, since the efficacy of enzymatic and nonenzymatic antioxidant mechanisms dramatically declines with age [18]. The main source of ROS production is oxidative phosphorylation during mitochondrial metabolism. Since mitochondria build up 45% of cardiomyocytes, the ROS they generate are of paramount importance [19]. Cardiac vulnerability is strongly linked to this aggravated oxidative injury, as it is responsible for the premature apoptosis of the cardiomyocytes, by damaging intracellular macromolecules [20]. Our results clearly show that aging arise an elevated cardiac ROS production both in males and females; however, 12 weeks of RESV administration was able to moderate the oxidative processes by scavenging free radicals. RESV is considered to be an impressive antioxidant pharmacophore thanks to its 4-hydroxystilbene skeleton. The antioxidant activity of RESV is in part attributed to the existence of its free hydroxyl group. Besides, it potentiates endogenous antioxidant enzymes such as SOD, GSH, or HO by the interaction of Nrf2 which is considered to be the main target of RESV. RESV facilitates the translocation of Nrf2 to the nucleus and triggers the transcription of antioxidant defense enzymes [21]. It has been previously reported that RESV upregulates the gene expression of HO enzymes in a Nrf2-dependent manner, along this exact pathway [22]. During the breakdown of red blood cells, HO catalyzes the degradation of heme, resulting in the formation of biliverdin, ferrous iron, and carbon monoxide (CO). Biliverdin, with the help of biliverdin reductase, is converted to bilirubin which has been shown to protect against oxidative mechanisms by reducing oxygen radicals, NADPH oxidase, and adhesion molecules [23]. Moreover, a recent research regarding HO activity attributes its antioxidant role not only to the bilirubin/biliverdin redox cycle but also to CO [24]. CO, derived from HO activity, is responsible for regulating the GSH system as well [25]. GSH is a tripeptide of three amino acids that is synthesized as a primary line of antioxidant defense. Its free -SH group is capable of binding metal ions, and as a substrate for glutathione peroxidase (GPx), it is involved in the reduction of H_2_O_2_ and lipid peroxides [26]. Interestingly, the findings of Ungvari et al. supported that RESV also increases cellular GSH content via Nrf2 activation [27]. Previous work by our research group has shown that HO and GSH systems are inseparable, and their coordinated function is essential for the proper function of cardiac cells [28]. Several studies have shown that the efficiency of the HO and GSH system declines dramatically with age, resulting in a deterioration of the cell's tolerance to oxidative stress [28, 29]. Similarly, we observed that HO and GSH values were diminished in aged groups for both sexes. Nonetheless, a prolonged RESV treatment intensified the antioxidant mechanisms by boosting the synergic HO activity and GSH system. Supporting our results, mounting evidence indicates that RESV augments cellular antioxidant capacity through the reduction of reactive oxygen species (ROS) level, in parallel with the increase of glutathione (GSH), heme oxygenase (HO), and superoxide dismutase (SOD) activity [9]. It is also important to note that changes in the redox state of the cells are causally related to the systematic inflammatory processes. In the 2000s, Claudio Franceschi puts forward an interesting hypothesis, namely, that ageing organisms tend to develop a chronic inflammatory state characterized by persistently high level of proinflammatory cytokines (TNF-*α*, IL-1, and IL-6) in tissues and cells [30]. In this context, several lifespan-affecting biochemical pathways have been discovered over the last decades, the vast majority of which are mediated through the activation of NF*κ*B signaling. NF*κ*B is an important dimeric transcription factor and plays a fundamental role in biological processes associated with ageing, including inflammation, cell survival, and stress response. The inflammatory state resulting from ageing-associated dysregulated NF*κ*B signaling is characterized by increased MPO activity, elevated C reactive protein (CRP), and TNF-*α* concentrations [31, 32]. Ageing, in fact, is a progressive spread of inflammatory processes, and it is now clear that it is one of the main risk factors for CVDs [33]. Our findings have also underpinned that in the heart of aging females and males, a severe inflammatory state was manifested as a result of increased TNF-*α* concentration and MPO activity due to the upregulation of the NF*κ*B pathway. However, 12 weeks of RESV-treatment contributed to the moderation of cardiac inflammation by decreasing MPO activity, the expression of TNF-*α* and NF*κ*B. Confirming our results, both in vivo and in vitro studies substantiated the anti-inflammatory properties of RESV trough the inhibition of inflammatory factors and pathways [34]. Previous studies verified that RESV suppresses NF*κ*B activation and gene expression along with the expression of proinflammatory cytokines [35]. According to Grujic Milanovic et al., RESV intake protected the cardiomyocytes through the inhibition of MPO activity, suggesting its promising anti-inflammatory and cardioprotective properties [36]. A remarkable finding from Yan et al. discussed that RESV improved cardiovascular function by decreasing circulating levels of proinflammatory cytokines such as of tumor necrosis factor-*α* (TNF-*α*) or interleukin-6 (IL-6) and by suppressing nuclear factor kappa B (NF-*κ*B) pathway [10]. Similarly, another study showed that RESV intake significantly reduced myocardial infarction areas together with myeloperoxidase (MPO) and TFN-*α* levels in the myocardium [11]. Along with the ability to decrease proinflammatory markers, RESV was observed to increase anti-inflammatory cytokines in the heart as well [37]. Maintaining a proper equilibrium between oxidant/antioxidant processes as well as between proinflammatory and anti-inflammatory agents provides the integrity of the body and the heart. In addition to the beneficial effects of RESV discussed in our study, it has proven to be cardioprotective in many other ways. RESV modulates the renin-angiotensin system and enhances the production of nitrogen monoxide (NO), thus proved to be effective in the pathomechanism of hypertension, atherosclerosis, or ischemic heart disease [38, 39]. Growing evidence support that RESV exerts its cardioprotective effect by reducing oxidative stress and inflammation, improving Ca^2+^ homeostasis and decreasing cardiomyocyte apoptosis [40]. Interestingly, Fourny et al. found that RESV presents high potential to reduce ischemia-reperfusion injury in rat heart [41]. To support the cardioprotective effects of RESV, we analyzed the extent of cardiac damage induced by an acute cardiac injury. Our findings demonstrated that the necrotic area of the hearts was significantly attenuated as a result of 3-month long RESV treatment in both sexes. In accordance with our results, Xi et al. also verified the RESV-induced cardioprotection against ischemia-reperfusion injury [42]. Based on our results and other consistent data, we can conclude that RESV exerts its cardioprotective actions through its ability to balance inflammatory and oxidative mediators (Figure 7). RESV is proved to be a promising bioactive compound in several aspects of healthcare research and should be considered as a good therapeutic strategy in cardiovascular fields.

## 5. Conclusion

RESV is one of the most widely studied bioactive compounds, not only for its anti-inflammatory and antioxidant effects but also due its apparent lack of toxicity. It is clear that RESV was able to alleviate the age-related adverse changes in the heart of female and male rats, thereby making the myocardium more resistant to ischemic injury. Hence, our observations indicate that RESV can be considered as a potential bioactive compound in the regulation of redox homeostasis and inflammatory responses concurrent with cardioprotection. Research on RESV focusing its distinct mechanisms connected to the mitigation of ageing-related oxidative and inflammatory processes and their pathological consequences could open up important preventive and therapeutic targets for CVD.

## Figures and Tables

**Figure 1:** The effects of a 12-week-long resveratrol treatment on the magnitude of the infarct size in aged rats. Infarct size (IS) was calculated as the percentage of the area at risk (AAR). One-way ANOVA and Tukey posttest result is shown as mean ± SD; *n* = 8 − 9/group, ^∗∗^*p* < 0.01, and ^∗∗∗∗^*p* < 0.0001. Statistical significance between resveratrol-treated and nontreated control counterparts. RESV: Resveratrol; IS: Infarct size; AAR: Area at risk.

**Figure 2:** (a) The effects of a 12-week-long resveratrol treatment on cardiac NF*κ*B concentration in aged rats (NF*κ*B; expressed as pg/mg protein). One-way ANOVA and Tukey posttest result is shown as mean ± SD; *n* = 7 − 8/group. (b) The effects of a 12-week-long resveratrol treatment on cardiac TNF-*α* expression in aged rats (TNF-*α*; expressed as pg/mg protein). One-way ANOVA and Tukey posttest result is shown as mean ± SD; *n* = 6 − 8/group. ^∗^*p* < 0.05, ^∗∗^*p* < 0.01, ^∗∗∗^*p* < 0.001, and ^∗∗∗∗^*p* < 0.0001: Statistical significance between resveratrol-treated and nontreated control counterparts. RESV: Resveratrol; NF*κ*B: Nuclear factor kappa B; TNF-*α*: Tumor necrosis factor alpha.

**Figure 3:** The effects of a 12-week-long resveratrol treatment on cardiac myeloperoxidase enzyme activity in aged rats (MPO; expressed as *μ*U/mg protein). Non-Gaussian distribution and Kruskal-Wallis test with Dunn's post hoc test result is shown as mean ± SD; *n* = 7 − 8/group. ^∗∗∗^*p* < 0.001: Statistical significance between resveratrol-treated and nontreated control counterparts. RESV: Resveratrol; MPO: Myeloperoxidase.

**Figure 4:** The effects of a 12-week-long resveratrol treatment on cardiac reactive oxygen species in aged rats (ROS; expressed as U/mg protein). Non-Gaussian distribution and Kruskal-Wallis test with Dunn's post hoc test result is shown as mean ± SD; *n* = 7 − 9/group and ^∗^*p* < 0.05: Statistical significance between resveratrol-treated and nontreated control counterparts. RESV: Resveratrol; ROS: Reactive oxygen species.

**Figure 5:** The effects of a 12-week-long resveratrol treatment on cardiac GSH+GSSG content in aged rats (GSH+GSSG; expressed as nmol/mg protein). Non-Gaussian distribution and Kruskal-Wallis test with Dunn's post hoc test result is shown as mean ± SD; *n* = 7 − 9/group and ^∗∗^*p* < 0.01: Statistical significance between resveratrol-treated and nontreated control counterparts. RESV: Resveratrol; GSH+GGSG: Total glutathione.

**Figure 6:** The effects of a 12-week-long resveratrol treatment on cardiac HO activity in aged rats (HO activity; expressed as nmol/bilirubin/h/mg protein). One-way ANOVA and Tukey posttest result is shown as mean ± SD; *n* = 7 − 8/group, ^∗∗^*p* < 0.01, and ^∗∗∗∗^*p* < 0.0001: Statistical significance between resveratrol-treated and nontreated control counterparts. RESV: Resveratrol; HO: Heme oxygenase.

**Figure 7:** Summary of the study. Resveratrol sufficiently suppressed the age-related inflammatory pathways including the expression of TNF-*α*, NF*κ*B, and the activity of MPO while intensified the endogenous antioxidant defenses through the induction of GSH and HO system. Presumably, as a result of these processes, the necrotic extension of the heart was also significantly reduced. HO: Heme oxygenase; GSH+GGSG: Total glutathione; ROS: Reactive oxygen species; NF*κ*B: Nuclear factor kappa B; TNF-*α*: Tumor necrosis factor alpha; MPO: Myeloperoxidase enzyme.

## Data Availability

All data used to support the findings of this study are included within the article.
